The article "Neuroprotective Effects of Curcumin against Oxygen-Glucose Deprivation/Reoxygenation-Induced Injury in Cultured Primary Rat Astrocyte by Improving Mitochondrial Function and Regulating the ERK Signaling Pathway" was published in 2022. Journal: Evid Based Complement Alternat Med.

# Neuroprotective Effects of Curcumin against Oxygen-Glucose Deprivation/Reoxygenation-Induced Injury in Cultured Primary Rat Astrocyte by Improving Mitochondrial Function and Regulating the ERK Signaling Pathway

**DOI:** 10.1155/2022/1731701

**Published:** 2022-07-12

**Authors:** Haojie Chen, Guoke Tang, Jiangming Yu, Ronghua Yu

**Affiliations:** ^1^Department of Orthopedics, Tongren Hospital, Shanghai Jiao Tong University School of Medicine, Shanghai 200336, China; ^2^Department of Orthopedics, Shanghai General Hospital, Shanghai Jiaotong University, No. 100 Haining Road, Shanghai 200080, China

## Abstract

**Objectives:**

Curcumin (Cur) is a natural polyphenol isolated from turmeric and has potent anti-inflammatory and antioxidant activities. This study aimed to explore the effects and possible mechanisms of curcumin on oxygen-glucose deprivation/reoxygenation (OGD/R)-induced injury in cultured rat astrocyte primary cells.

**Methods:**

After screening for effective doses, the cultured rat astrocyte primary cells were divided into three groups: control, OGD/R, and OGD/R + curcumin (10 *μ*M, 20 *μ*M, and 40 *μ*M). Cell viability was detected using CCK8 assays. The level of malondialdehyde and superoxide dismutase activity was determined using commercial kits. The endothelial nitric oxide synthase and adenosine triphosphate concentrations were determined by enzyme-linked immunosorbent assay. The mRNA levels of the inflammatory indexes interleukin (IL)-6, tumor necrosis factor (TNF)-alpha, and interleukin (IL)-1*β* were evaluated by quantitative reverse-transcription polymerase chain reaction. Annexin V-fluorescein isothiocyanate/propidium iodide was used to detect apoptosis. JC-1 was used to assess the mitochondrial membrane potential. The protein expression of apoptosis-related proteins (B-cell lymphoma-2 (Bcl-2), BCL-2-associated X (Bax), and cleaved caspase 3), mitochondria-related proteins (dynamin-related protein 1 (DRP1), phosphorylated DRP1 (p-DRP1), and mitofusin 2), and essential proteins of the extracellular signal-regulated kinase (ERK) signaling pathway (ERK1/2, p-ERK1/2) were analyzed by western blot.

**Results:**

Our data indicated that curcumin reversed OGD/R-induced cell viability loss, oxidative stress, inflammatory cytokine production, and cell apoptosis in a dose-dependent manner. Furthermore, curcumin attenuated OGD/R-induced mitochondrial dysfunction and ERK1/2 phosphorylation in a dose-dependent manner.

**Conclusions:**

Curcumin protected against OGD/R-induced injury in rat astrocyte primary cells through improving mitochondrial function and regulating the ERK signaling pathway.

## 1. Introduction

Spinal cord injury (SCI) is a devastating problem that leads to sensory and functional disabilities in some of the body's internal organs below the level of the injury [1]. The original spinal cord injury is a primary damage that triggers secondary injury [2]. Secondary injury produces a cascade of biochemical, mechanical, and physiological changes, leading to further spinal cord damage [3]. Secondary injury plays a pivotal role in the final prognosis and is a potential therapeutic target for the management of SCI [4]. Astrocytes are the most common glial cells that provide metabolic support to the central nervous system (CNS) [5]. Astrocyte dysfunction can amplify neuroinflammation and cause further injury to neurons [6]. Mitochondria, where bio-oxidation and energy generation occur, are essential organelles for cell survival [7] and are also susceptible to injuries [8]. Acute SCI can induce morphological and functional changes in astrocytic mitochondria, which are closely related to the pathogenesis of secondary SCI [9]. The extracellular signal-regulated kinase (ERK)/dynamin-related protein 1 (DRP1) signaling pathway mediates mitochondrial dysfunction during secondary SCI injury [10, 11].

Curcumin (Cur), a hydrophobic polyphenol derived from the dried rhizomes of *Curcuma longa* L. (turmeric), has long been used in traditional Chinese medicine [12]. It was initially used as a cooking spice in some Asian countries [13] and has received a great deal of attention for the therapy of several diseases, including cardiovascular disease [14], cancer [15], and conditions of the CNS [16]. As a natural product, curcumin has been shown to have potent anti-inflammatory and antioxidant activities, which are closely related to its therapeutic effects [17]. It also plays a protective role in SCI [18–20]. However, the underlying mechanisms of curcumin in the treatment of SCI are not entirely understood.

In the present study, we explored the effects of curcumin on primary rat astrocyte damaged by oxygen-glucose deprivation/reoxygenation (OGD/R) and its possible mechanism of action on mitochondrial function and the ERK signaling pathway.

## 2. Methods

### 2.1. Astrocyte Culture

All animals were treated according to the National Institutes of Health guidelines for the Care and Use of Laboratory Animals. Primary spinal cord astrocyte was isolated from six newborn Sprague Dawley rats, as previously described [21]. Briefly, the newborn rats were deeply anesthetized with isoflurane and then decapitated. The spinal column was cut and placed on ice in a glass culture dish. The spinal cord above the T10 level was removed with sterile phosphate-buffered saline (PBS). Spinal cord tissues were cut into small pieces and digested with 0.125% trypsin. The mixture was filtered with 70 *μ*m sterile sieves and placed in a complete DMEM/high-glucose medium (^#^SH30022.01, Hyclone, USA) containing 10% fetal bovine serum (^#^10270-106, fetal bovine serum, Gibco, USA). Cells were incubated at 37°C with 5% CO_2_ for five days, and then the mixed microglial cells and oligodendrocytes were removed by shaking at 37°C overnight at 200 rpm.

### 2.2. OGD/R Protocol

The cultured rat astrocyte primary cells were washed three times with PBS and incubated with serum-free DMEM. Then, the cells were placed in an anaerobic environment (1% O_2_, 5% CO_2_, and 94% N_2_) at 37°C for 6 h, namely, OGD. Astrocytes were washed once with PBS after 6 h of OGD and placed in the normal conditions (reoxygenation) and complete DMEM culture with 10% BSA.

### 2.3. CCK8

The isolated astrocyte was seeded in a 96-well plate at a density of 8,000 cells per well and incubated at room temperature overnight. Curcumin (^#^C110685, Aladdin, China) was added at various concentrations (1 *μ*M, 5 *μ*M, 10 *μ*M, 20 *μ*M, and 40 *μ*M) into the medium 30 min before OGD and at the time of reoxygenation. Approximately 24 h after oxygen-glucose deprivation/reoxygenation (OGD/R), 10 mL of CCK8 solution (^#^CA1210, Solarbio, China) was added and incubated in the dark for 1 h. The optical density values were measured at a wavelength of 450 nm.

### 2.4. Immunofluorescence Staining

The astrocyte was grown on coverslips overnight and then fixed with 4% paraformaldehyde. Cells were permeabilized with 0.3% Triton X-100 and blocked with 10% BSA. Astrocyte was incubated individually with astrocytic markers (GFAP and S100*β*) and antibodies (^#^PAB32097 and ^#^ PAB30176, Bioswamp, China) at 4°C overnight. Then, fluorescein isothiocyanate (FITC, red) or Alexa Fluor 488 (green)-conjugated secondary antibodies were added. The protein expression of GFAP and S100*β* was observed using a fluorescence microscope (Leica, Germany).

### 2.5. Oxidative Stress Indexes

The malondialdehyde (MDA) and superoxide dismutase (SOD) levels were detected by using MDA and SOD commercial kits (^#^A003-1-1 and ^#^A001-3-2; Nanjing Jiancheng Bioengineering Institute, China) by following the manufacturer's manuals.

### 2.6. Enzyme-Linked Immunosorbent Assay (ELISA)

Endothelial nitric oxide synthase (eNOS) and adenosine triphosphate (ATP) concentrations were detected by rat eNOS and ATP ELISA kits (^#^RA20010 and ^#^RA20768, Bioswamp, China) by following the manufacturer's manuals.

### 2.7. Reactive Oxygen Species (ROS) Production Assay

The intracellular ROS levels were determined with a commercial ROS kit (^#^S0033, Beyotime, China) by following the manufacturer's manuals. After treatment of curcumin and OGD/R for 24 h, astrocyte was incubated with 2′-7′-dichlorofluorescein diacetate. After washing, the cells were suspended in PBS, and the fluorescence was detected by flow cytometry (ACEA Biosciences, USA).

### 2.8. Quantitative Reverse-Transcription Polymerase Chain Reaction (qRT-PCR)

The total RNA was extracted by RNA isoPlus (^#^KM4101, KAPA Biosystems, USA) according to the manufacturer's instructions. Total RNA (500 ng) was reverse-transcribed to obtain cDNA. The forward and reverse primers were as follows: 5′-TGGAGTTCCGTTTCTACCTGG-3′ and 5′-GGATGGTCTTGGTCCTTAGCC-3′ for the interleukin (IL)-6 gene; 5′-CCACGCTCTTCTGTCTACTG-3′ and 5′-GAAAGCCCTGTA-3′ for tumor necrosis factor-alpha (TNF-*α*); 5′-CAAGCAACGACAAAATCCC-3′ and 5′-CAAACCGCTTTTCCATCTTC-3′ for IL-1*β* gene; and 5′-CGTTGACATCCGTAAAGAC-3′ and 5′-TAGGAGCCAGGGCAGTA-3′ for the internal control *β*-actin gene.

### 2.9. Annexin V-FITC Flow Cytometry

The early cell apoptosis was detected by Annexin V-FITC/propidium iodide (PI) apoptosis detection kit (^#^556547, BD Biosciences, USA). The procedure for curcumin treatment and OGD/R modeling was the same as described above. The cells were washed twice after all groups of cells were harvested. Annexin V-FITC and PI were added by following the manufacturer's protocols. The cell apoptosis was determined by flow cytometry (ACEA Biosciences, USA).

### 2.10. Western Blotting

Cell lysates used for electrophoresis were collected from all cell groups. Western blot analysis was performed as previously indicated [22]. Primary antibodies for the subsequent experiments are as follows: rabbit anti-B-cell lymphoma 2 (Bcl-2) antibody (^#^PAB44408, Bioswamp, China), rabbit anti-BCL-2-associated X (Bax) antibody (^#^PAB30861, Bioswamp, China), rabbit anti-cleaved caspase 3 antibody (^#^ab49822, Abcam, USA), rabbit anti-dynamin-related protein 1 (DRP1) antibody (^#^PAB33409, Bioswamp, China), rabbit anti-phosphorylated DRP1 (p-DRP1) (s637) antibody (^#^4867S, CST, USA), rabbit anti-mitofusin 2 (MFN2) antibody (^#^PAB37988, Bioswamp, China), rabbit anti-ERK antibody (^#^PAB37123, Bioswamp, China), rabbit anti-phosphorylated ERK (p-ERK) antibody (^#^4370T, CST, USA), and rabbit anti-*β*-actin antibody (^#^PAB36265, Bioswamp, China). Then cells were incubated with the appropriate secondary antibodies, and signals were detected by the automatic imaging system (Tanon-5200, Tanon, China).

### 2.11. Mitochondrial Membrane Potential Detection

The mitochondrial membrane potential (ΔΨm) was detected by JC-1 detection kit (^#^C2006; Beyotime, China) according to the supplier's protocol. In brief, astrocyte in all groups was stained with JC-1, which presented potential-dependent aggregation in mitochondria. JC-1 exhibits green fluorescence (527 nm) at low membrane potential while producing red fluorescence (590 nm) at high membrane potential.

### 2.12. Transmission Electron Microscopy

The astrocyte cells were digested and centrifuged. Then, the cells were collected and fixed with 2.5% glutaraldehyde and 1% osmic acid. After dehydration, the cells were embedded in epoxy resin. The cell slices were stained with 2% uranyl acetate and lead citrate. The cellular mitochondria were observed with a transmission electron microscope (TEM; Hitachi HT7700, Japan).

### 2.13. Statistical Analysis

The results are expressed as mean ± standard deviation. The differences among groups were analyzed by one-way analysis of variance. The statistical significance was established at *P* < 0.05. Statistical analysis was performed by the SPSS software. The graphs were produced by using GraphPad Prism software.

## 3. Results

### 3.1. Purity Identification of Isolated Primary Rat Astrocyte

Immunofluorescence staining of astrocytic markers (GFAP and S100*β*) was performed to determine the purity of the astrocyte. After 24 h of incubation, cells were uniformly stained with anti-GFAP and anti-S100*β* antibodies. The high purity of isolated primary rat astrocyte is shown in Figures 1(a) and 1(b).

### 3.2. Screening for Effective Concentration of Curcumin against OGD/R Injury in Astrocyte

The cell viability of cultured astrocyte was determined through CCK8 assay, which was used to evaluate the protective effects of curcumin against OGD/R-induced cytotoxicity. Compared to the control group, there is a significant reduction in cell viability in the OGD/R group, which was restored by curcumin pretreatment (1, 5, 10, and 20 *μ*M) in a dose-dependent way (Figure 2).

### 3.3. Curcumin Pretreatments Attenuated Loss of Cell Viability and Increased Oxidative Stress Indexes in Rat Astrocyte Primary Cells Injured with OGD/R

Cell viability and oxidative stress indices were investigated to evaluate the protective effects of curcumin on rat astrocyte primary cells injured by OGD/R. The results showed that the pretreatments with curcumin (10, 20, and 40 *μ*M) increased cell viability after exposure in a dose-dependent way (Figure 3(a)). The intracellular concentrations of MDA, SOD, eNOS, and ROS were determined to evaluate the antioxidative effects of curcumin. In OGD/R group, the MDA concentration was increased significantly, but markedly reduced by pretreatment with curcumin (10, 20, and 40 *μ*M) (Figure 3(b)). SOD activity and eNOS levels decreased after OGD/R exposure, which was restored by pretreatment with curcumin (10, 20, and 40 *μ*M) (Figures 3(c) and 3(d)). Additionally, ROS levels were significantly elevated after exposure to OGD/R, and curcumin pretreatment reduced ROS production in the dose-dependent way (Figure 3(e)).

### 3.4. Curcumin Pretreatments Inhibited Inflammatory Responses in OGD/R-Injured Primary Rat Astrocyte

To assess the curcumin effects on OGD/R-induced inflammatory responses in rat astrocyte, intracellular mRNA concentrations of IL-6, TNF-*α*, and IL-1*β* were measured. The data indicated that the elevated mRNA concentrations of IL-6, TNF-*α*, and IL-1*β* following OGD/R injury were reduced with curcumin (10 *μ*M, 20 *μ*M, and 40 *μ*M) pretreatment in the dose-dependent way (Figures 4(a)–4(c)).

### 3.5. Curcumin Pretreatments Inhibited Cell Apoptosis in OGD/R-Injured Rat Astrocyte Primary Cells

The rate of apoptosis and the expression of apoptosis-related proteins (Bax, Bcl-2, and cleaved caspase 3) were detected to evaluate the curcumin effects on OGD/R-induced cell apoptosis in rat astrocyte primary cells. The apoptosis rate was observably elevated in OGD/R group, while the curcumin pretreatment alleviated the apoptosis (Figures 5(a) and 5(b)). Western blot assay revealed that OGD/R-induced cell apoptosis was concomitant with increased expression of Bax and cleaved caspase 3 and decreased expression of Bcl-2 in cultured rat astrocyte primary cells. Apoptosis was reversed through pretreatment with curcumin (10 *μ*M, 20 *μ*M, and 40 *μ*M) in the dose-dependent way (Figures 5(c)–5(g)).

### 3.6. Curcumin Pretreatments Alleviated Mitochondrial Damage in OGD/R-Injured Primary Rat Astrocyte

The degree of mitochondrial depolarization in cultured astrocyte was evaluated by JC-1. After exposure to OGD/R, the ΔΨm of astrocyte increased, which was reduced by pretreatment with curcumin (10, 20, and 40 *μ*M) (Figures 6(a) and 6(b)). The results showed that ATP production decreased significantly in the OGD/R group, whereas curcumin (10, 20, and 40 *μ*M) pretreatment restored ATP production (Figure 6(c)). The expression of mitochondrial-related proteins (DRP1, p-DRP1, and MFN2) was detected to evaluate mitochondrial function. DRP1 expression was significantly increased in the OGD/R group and decreased by curcumin (10, 20, and 40 *μ*M) pretreatment. The presentation of p-DRP1 and MFN2 was markedly reduced in the OGD/R group, which was restored by pretreatment with curcumin (10, 20, and 40 *μ*M) (Figures 6(d)–6(g)). In the OGD/R group, mitochondrial swelling and loss of cristae were observed using a TEM, while pretreatment with curcumin (10, 20, and 40 *μ*M) attenuated these morphological changes in mitochondria (Figure 6(h)).

### 3.7. Curcumin Pretreatments Regulated the ERK1/2 Signaling Pathway in OGD/R-Injured Primary Rat Astrocyte

The ERK1/2 signaling pathway is critical for astrocyte survival [23]. The results revealed that the ERK1/2 phosphorylation increased in the OGD/R group, which was reduced through pretreatment with curcumin (10 *μ*M, 20 *μ*M, and 40 *μ*M) in a dose-dependent way (Figures 7(a)–7(c)).

## 4. Discussion

SCI, an incurable disease, often results in devastating sequelae [24]. Astrocytes are the most abundant glial cells in the central nervous system (CNS) and have been known to protect neurons and assist their survival under pathological conditions [25]. Astrocyte dysfunction contributes to the secondary injury in SCI [26]. Therefore, astrocyte may be potential targets for SCI therapy. Curcumin was reported to be effective in treating SCI [19, 27]. Curcumin's therapeutic effects have been closely related to its own anti-inflammatory and antioxidant activities [28], although the potential mechanisms are still only partly understood. The present study demonstrates that curcumin exerts potent antioxidant, anti-inflammatory, and neuroprotective effects on primary rat astrocyte damaged by OGD/R. These effects are mediated by improving mitochondrial function and regulating the ERK signaling pathway.

Mitochondria produce ATP, which is essential for cell viability [29]. Mitochondria are also vulnerable to various injuries [30]. Dysfunction of astrocytic mitochondria can cause deleterious actions on neurons via astrocyte-neuron interactions [31]. Mitochondria have emerged as potential therapeutic targets for treating SCI [30]. DRP1 is a key protein that promotes mitochondrial fission [32]. Excessive mitochondrial fission is correlated with DRP1 dephosphorylation at Ser 637, resulting in mitochondria morphological changes [32]. MFN2, a dynamin-like GTPase, is involved in mitochondrial fusion [33]. The absence of MFN2 leads to mitochondrial fragmentation and neurodegeneration [34]. Curcumin pretreatment not only attenuated mitochondrial swelling and loss of cristae in injured astrocyte induced by OGD/R, but also improved DRP1 phosphorylation in Ser 637 and MFN2 expression in the current study. The findings are consistent with the results of previously published studies [32, 35, 36].

ERK is essential for the regulation of cell proliferation, differentiation, and survival [37], and its signaling pathway which is closely related to mitochondrial function and cell viability [38, 39] is critical to the survival of astrocyte [40]. ERK phosphorylation is elevated after SCI [22], and overactivation of the ERK signaling pathway is involved in persistent inflammation and neuropathic pain sequela [41]. In this study, ERK phosphorylation was increased in the OGD/R group, while curcumin pretreatment decreased p-ERK expression.

In conclusion, curcumin protects against OGD/R-induced injury in rat astrocyte primary cells through improving mitochondrial function and regulating the ERK signaling pathway.

## Figures and Tables

**Figure 1:** Purity identification of isolated primary astrocyte. (a, b). Representative immunofluorescence images showing the purity of isolated primary astrocyte by GFAP and S100*β* (×200). The representative images are from three independent experiments.

**Figure 2:** Screening for an effective concentration of curcumin against oxygen-glucose deprivation/reoxygenation (OGD/R). The effective concentration of curcumin against OGD/R was determined by CCK8 assay; versus control group, ^*∗*^*P* < 0.05, ^*∗∗*^*P* < 0.01, ^*∗∗∗*^*P* < 0.001, respectively; versus OGD/R group, ^#^*P* < 0.05, ^##^*P* < 0.01, and ^###^*P* < 0.001. (*n* = 3). OD = optical density.

**Figure 3:** Curcumin pretreatments alleviated loss of cell viability and increased oxidative stress induced by oxygen-glucose deprivation/reoxygenation (OGD/R) in primary rat astrocyte. (a) Summary of data presenting astrocyte proliferation using the CCK8 test. (b, c) Summary of data presenting intracellular malondialdehyde (MDA) concentrations and superoxide dismutase (SOD) levels with commercial kits. (d) Summary of data presenting intracellular endothelial nitric oxide synthase (eNOS) level by enzyme-linked immunosorbent assay (ELISA) kits. (e) Summary of data presenting intracellular reactive oxygen species (ROS) production with flow cytometry. Versus control group, ^*∗*^*P* < 0.05, ^*∗∗*^*P* < 0.01, ^*∗∗∗*^*P* < 0.001, respectively; versus OGD/R group, #*P* < 0.05, ^##^*P* < 0.01, and ^###^*P* < 0.001. (*n* = 3). OD = optical density.

**Figure 4:** Curcumin pretreatments inhibited inflammatory responses induced by oxygen-glucose deprivation/reoxygenation (OGD/R) in rat astrocyte. (a) The mRNA level of interleukin-6 (IL-6). (b) The mRNA level of tumor necrosis factor-alpha (TNF-*α*). (c) The mRNA level of IL-1*β*. Versus control group, ^*∗*^*P* < 0.05, ^*∗∗*^*P* < 0.01, ^*∗∗∗*^*P* < 0.001, respectively; versus OGD/R group, ^#^*P* < 0.05, ^##^*P* < 0.01, and ^###^*P* < 0.001 (*n* = 3).

**Figure 5:** Curcumin pretreatments inhibited cell apoptosis in oxygen-glucose deprivation/reoxygenation (OGD/R)-injured astrocyte. (a) The apoptosis ratio evaluated by Annexin V/propidium iodide (PI) assay. (b) Summary of data showing changes in apoptosis ratio. (c–g) Representative images and summary of data for relative protein expressions of BCL-2-associated X (Bax), B-cell lymphoma 2 (Bcl-2), and cleaved caspase 3 through western blot analysis. Versus control group, ^*∗*^*P* < 0.05, ^*∗∗*^*P* < 0.01, ^*∗∗∗*^*P* < 0.001, respectively; versus OGD/R group, ^#^*P* < 0.05, ^##^*P* < 0.01, and ^###^*P* < 0.001 (*n* = 3).

**Figure 6:** Curcumin pretreatments alleviated mitochondria damage in oxygen-glucose deprivation/reoxygenation (OGD/R)-injured astrocyte. (a) Flow cytometry detection of alterations in JC-1 (fluorescence color reflecting alterations in the mitochondrial membrane potential). (b) Summary of data of the alterations of mitochondrial membrane potential. (c) Summary of data showing levels of intracellular adenosine triphosphate (ATP). (d–g) Representative images and summarized data for relative protein expressions of phosphorylated dynamin-related protein 1 (p-DRP1; Ser 637), DRP1, and mitofusin 2 (MFN2) by western blot analysis. (h) Representative images of transmission electron microscopy of astrocytic mitochondria. Versus control group, ^*∗*^*P* < 0.05, ^*∗∗*^*P* < 0.01, ^*∗∗∗*^*P* < 0.001, respectively; versus OGD/R group, ^#^*P* < 0.05, ^##^*P* < 0.01, and ^###^*P* < 0.001 (*n* = 3).

**Figure 7:** Curcumin pretreatments regulated the ERK1/2 signaling pathway in oxygen-glucose deprivation/reoxygenation (OGD/R)-injured astrocyte. (a) Representative images of the phosphorylated extracellular signal-regulated kinase (p-ERK) and ERK protein expressions by western blotting. (b, c) Summary of data for relative protein expressions of p-ERK to ERK and ERK to *β*-actin.

## Data Availability

The data sets used and/or analyzed in the study are available from the corresponding author on reasonable request.
